The article "The stem cell factor antibody enhances the chemotherapeutic effect of adriamycin on chemoresistant breast cancer cells" was retracted in 2013. Reasons: errors in the methods; errors in the results or conclusions.

# The stem cell factor antibody enhances the chemotherapeutic effect of adriamycin on chemoresistant breast cancer cells

**DOI:** 10.1186/1475-2867-12-21

**Published:** 2012-05-29

**Authors:** Neil D Jelly, Issam I Hussain, Jennifer Eremin, Oleg Eremin, Mohamed El-Sheemy

**Affiliations:** 1 University of Lincoln, Brayford Pool, Lincoln, LN6 7TS, UK; 2 Research & Development, Lincoln County Hospital, Greetwell Road, Lincoln, LN2 5QY, UK; 3 Queens Medical Centre, University of Nottingham, Derby Road Nottingham, Nottingham, NG7 2UH, UK

## Abstract

**Background:**

The outcome of chemotherapy in breast cancer is strongly influenced by multidrug resistance (MDR). Several surrogate markers of chemoresistance have been identified including - CD24 (cluster differentiation 24) expression, stem cell growth factor (SCF), B-cell lymphocyte protein 2 (Bcl-2) and annexin V. The present study aimed to examine the expression of CD24 in the sensitive breast cancer cell line MCF-7 (Michigan Foudation-7) and MCF-7/adriamycin resistant (MCF-7/AdrRes) cells, and, if minimal effective doses of the anthracycline drug adriamycin (0.579 μM and 88.2 μM) would be enhanced by the antibody to SCF (anti-SCF).

**Methods:**

CD24 expression was analysed by flow cytometry. Both Bcl-2 and annexin V protein expression were quantitatively assessed by the enzyme-linked immunosorbent assay (ELISA).

**Results:**

In MCF-7/AdrRes cells the expression of CD24 was significantly higher compared to MCF-7 cells, 86.6% and 16.3% (p < 0.001), respectively. Bcl-2 expression was significantly increased in the presence of adriamycin and SCF (p < 0.038) and decreased in the presence of adriamycin and anti-SCF. When adriamycin, anti-SCF and SCF were combined or when adriamycin was used alone the decrease in Bcl-2 expression was insignificantly altered. In the presence of both adriamycin and SCF the expression of annexin V was decreased. However, it was significantly increased in the presence of adriamycin and anti-SCF (p < 0.042), as well as adriamycin, anti-SCF and SCF combined.

In MCF-7 cells the effect of adriamycin alone or with either SCF, anti-SCF or anti-SCF or SCF combined, did not significantly alter the expression of Bcl-2. However, in the presence of both adriamycin and SCF the expression of annexin V was decreased, but was significantly increased in the presence of adriamycin and anti-SCF (p < 0.001), adriamycin, anti-SCF and SCF combined and adriamycin alone. Our results demonstrate that anti-SCF with low dose of adriamycin reduces Bcl-2 expression in MCF-7/AdrRes cells and increases annexin V expression in both MCF7/AdrRes and MCF-7 cells.

**Conclusion:**

Adding anti-SCF to the chemotherapeutic regime of adriamycin may strongly enhance its chemotherapeutic effect in the treatment of patients with breast cancer.

## Introduction

Breast cancer is the most common form of cancer and the principal cause of death from cancer among women worldwide [1] Neoadjuvant chemotherapy (NAC) is frequently used to treat breast cancer patients particularly those with locally advanced disease in order to downstage and downgrade the disease [2] However, a complete pathological response is only observed in 30% of patients, whilst 70% of patients show an incomplete or no pathological response [3-7] Despite advances in understanding the molecular basis of breast cancer the poor responses to chemotherapeutic agents are not well defined. Several factors are attributed to drug resistance including - drug efflux, cancer stem cells (CSCs), cytokine overexpression and resistance to drug-induced apoptosis [8,9]. The ability to predict the response to NAC may result in a more cost-effective therapy. Therefore, targeting therapy to these potential responders would also avoid significant and unnecessary morbidity in nonresponders [3]. Adriamycin is an important drug component in NAC regimens however; breast cancer cells often become resistant to its effects. Critical apoptotic pathways, which are initiated by adriamycin and other cytotoxic drugs, are altered by several mechanisms resulting in chemoresistance. The ability to evade programmed cell death is a phenotypic characteristic of most tumours [10]. Negative regulators of apoptosis are amongst the most frequently studied particularly the proto-oncogene Bcl-2. Both B-cell lymphocytes and CSCs are characterised by extracellular protein expression of CD24, which may have an important role in both tumour growth and resistance. Nonetheless, it is thought that cancer stem cells (CSCs) are involved in carcinogenesis, local invasion and metastasis which play a key role to both radiotherapy and chemotherapy resistance [9]. Also, SCF may be co-expressed with Bcl-2 however their relationship requires further definition. Recently, an antibody to SCF (anti-SCF) significantly enhanced the cytotoxic effects of chemotherapy in human resistant haematological cancer [11]. However, it is not known whether anti-SCF enhances cytotoxicity in solid cancer e.g. breast cancer. On developing new molecular therapeutics understanding pharmacodynamic endpoints is critical. One of the characteristics of apoptosis is the externalization of phosphatidylserine (PS). It is documented that Annexin V is able to bind with high specificity to PS [12]. Therefore, the aim of this study was to evaluate the expression of CD24, and the ability of anti-SCF to enhance adriamycin by examining their combined effects on both Bcl-2 and annexin V expression in MCF-7 and MCF-7/AdrRes breast cancer cells.

## Materials and methods

### Cell culture of MCF-7 and MCF-7/AdrRes cell lines

The MCF-7 and MCF-7/AdrRes human breast adenocarcinoma cell lines were a kind gift from Queens Medical Centre, University of Nottingham, UK [3,9]. The MTT 3(4, 5 Dimethylthiazol-2-yl)-2,5-Diphenyltetrazolium Bromide) assay was used to establish minimal effective dose concentrations of adriamycin. In MCF-7/AdrRes cells the IC50 concentration for adriamycin was 88.2 μM versus 0.579 μM in MCF-7 cells. The cells were grown in tissue culture medium (TCM) consisting of RPMI-1640 (with L-glutamine) (Sigma Aldrich, UK), supplemented with 10% foetal calf serum (FCS) (Sigma Aldrich, UK), and 100 units/ml of penicillin/and 0.1- mg/ml of streptomycin (Sigma Aldrich, UK), and placed in an incubator. The incubator was set at 0.05 CO2 and humidified at 37°(C) throughout the study. All cells used subsequently in this study were between 15–20 passages. 2.2 Immunophenotyping for CD24 Expression Using Flow Cytometry Cultured cells were resuspended (0.5 × 10^6^ cells) in ice cold Phosphate Buffered Saline (PBS) and 10% FCS. Cells (0.5 × 10^6^) were then incubated for 30 minutes (mins) at 4°C with primary CD24 fluorescein isothiocyanate (FITC) murine monoclonal antibody (MoA) (Cambridge Biosciences, Cambridge, UK), which was prepared by diluting in 3% bovine serum albumin (BSA) and PBS (BSA/PBS) to a final concentration of 1 in 20. Cells were washed in PBS centrifuged at 300 g for 5 mins and resuspended in 500μls of ice cold PBS with 10% FCS for analysis by the Epics xL flow cytometer (Beckman Coulter, High Wycombe, UK) which was equipped with a standard argon laser for 488 nm excitation and with 525 nm band pass (FL1), 575 nm band pass (FL2), 620 nm band pass (FL3) and 675 nm band pass (FL4) filters.

### Treatment of MCF-7 and MCF-7/AdrRes cells

MCF-7 and MCF-7/AdrRes cell lines were cultured (5 × 10^3^ cells perwell) and were treated with adriamycin (Sigma Aldrich, UK) using 0.579 μM and 88.2 μM, respectively, to be effective in accordance with IC50 concentrations, 0.4 μg/ml anti-SCF (PeproTech EC LTD, UK), and/or 100 units/ml of SCF (0.4 μg/ml of anti-SCF fully inhibits the biological activity of SCF as previously established by our colleagues) [11]. The final concentration of 100 μl/well of treatment was incubated with the cells using the following parameters: (1) adriamycin with SCF; (2) adriamycin with anti-SCF; (3) adriamycin with both SCF and anti-SCF; (4) adriamycin alone. Cells were treated without adriamycin using the same parameters. Five replicates of each treated culture (2.5 × 10^4^ cells) were set and incubated for 48hs.

### Analysis of bcl-2 using the quantitative ELISA assay

The human Bcl-2 ELISA kit (Bender Med SystemsTM) was used to quantitatively analyse Bcl-2 protein, as described previously [11]. Cells were washed twice with PBS and centrifuged at 500 g for 5 mins. The cell pellets were resuspended at 5 × 10^6^/ml of lysis buffer for 60 mins at room temperature (RT). Cells were re-centrifuged and resuspended in sample diluent (serum matrix, buffered solution) 1:5. Each sample of cell lysate and lyophilized standards of serially diluted Bcl-2 (100μls) were duplicated and added with FITC-labelled biotin-conjugate (anti-Bcl-2 murine MoA) diluted 1:100 in the assay buffer (PBS, with 1% Tween 20 and 10% BSA), and incubated in a 96-microwell plate coated with murine MoA of human Bcl-2 for 2hs at RT. Using wash buffer (PBS containing 1% Tween 20) the microwell strips were thoroughly washed. Streptavidin-horseradish peroxidase (HRP) - conjugate was then added to all wells at a dilution of 1:100 in the assay buffer and incubated for 1 h at RT. Microwell strips were thoroughly washed again and then TMB substrate solution (1 × tetramethylbenzidine added to 1 × 0.02% - buffered hydrogen peroxide) was added for 10 mins and incubated at RT. The change in colour from the substrate reaction was monitored and was terminated by adding stop solution (1 M phosphoric acid). The absorbance of each microwell was then read at 450 nm using an ELISA plate reader (BMG Lab Technologies, Germany).

### Analysis of annexin V using the quantitative ELISA assay

The human annexin V ELISA kit (Bender Med SystemsTM) was used to quantitatively analyse annexin V protein, as previously reported [11]. Cells were washed twice with PBS and centrifuged at 500 g for 5 mins. The cell pellets were re suspended in sample diluent (serum matrix, buffered solution) (1:2). Each sample and lyophilized standards of serially diluted annexin V (100μls) were duplicated and added with FITC-labelled biotin-conjugate (anti-annexin V murine MoA) diluted 1:100 in the assay buffer (PBS, with 1% Tween 20 and 10% BSA). Samples were then incubated in a 96-microwell plate coated with murine MoA of human annexin V for 2hs at RT. Using wash buffer, (PBS containing 1% Tween 20) the microwell strips were washed thoroughly. Then at a dilution of 1:200 in the assay buffer, streptavidin-horseradish peroxidase (HRP) - conjugate was added to all wells and incubated for 1 h at RT. Microwell strips were again washed thoroughly with wash buffer with TMB substrate solution (1 × tetramethylbenzidine added to 1 × 0.02% - buffered hydrogen peroxide) then being added for 10 mins at RT. The change in colour from the substrate reaction was monitored and was terminated by adding stop solution (1 M phosphoric acid). The absorbance of each microwell was read at 450 nm using the ELISA plate reader (BMG Lab Technologies, Germany).

### Statistical analysis

The mean ± standard error of all readings underwent statistical analysis, whenever appropriate. Independent two-sample, two-tailed tests were used to analyse the difference in mean values of CD24 expression. Multi-factorial (three way) Analysis of Variance (ANOVA) was used to analyse the two response variables of Bcl-2 and annexin V. Statistical significance is recorded when the p-value was less than 0.05 (P < 0.05).

## Results

### CD24 expression

CD24 expression was measured by flow cytometry in MCF-7/AdrRes and MCF-7 cell lines (Figures 1 and 2). Levels of CD24 expression ranged from 86.6 ± 3.0% in resistant cells, compared with 16.3 ± 1.9% in wild type cells which was highly significant (p < 0.001).

**Figure 1:** **Expression of CD24 in MCF-7/AdrRes cells. Cells (10**^**4**^**) were analysed by flow cytometry using CD24 monoclonal antibody (FITC)**. The histogram shows high level expression for CD24 in cells (positives - 87%). Both the plots of forward scatter (FSC) versus side scatter (SSC) were used to gate cells (not shown). To show positivity of CD24 an (FL1) plot was used (shown). For the Epics xL flow cytometer λ excitation = 488 nm and λ emission = 525 nm.

**Figure 2:** **Expression of CD24 in MCF-7 cells**. Cells (10^4^) were analysed by flow cytometry using CD24 monoclonal antibody (FITC). The histogram shows low level expression for CD24 in cells (positives - 16%). Both the plots of forward scatter (FSC) versus side scatter (SSC) were used to gate cells (not shown). To show positivity of CD24 an (FL1) plot was used (shown). For the Epics xL flow cytometer λ excitation = 488 nm and λ emission = 525 nm.

### Effect of adriamycin/anti-SCF on bcl-2 expression in MCF-7/AdrRes and MCF-7 cells

The therapeutic effects of adriamycin, anti-SCF and SCF on Bcl-2 expression were examined by ELISA in MCF-7 and MCF-7/AdrRes cells, after being treated simultaneously for 48 hrs. The combination of adriamycin and SCF significantly increased Bcl-2 expression in MCF-7/AdrRes cells (p < 0.038), with a decrease in Bcl-2 expression observed after treatment with adriamycin and anti-SCF, adriamycin and both SCF and anti-SCF combined and adriamycin alone (Figure 3). In MCF-7 cells there was no significant difference in Bcl-2 expression observed after treatment with either adriamycin and SCF or adriamycin and anti-SCF, unlike in MCF-7/AdrRes cells. Similarly, no significant difference in Bcl-2 expression was observed in cells after treatment with adriamycin and both anti-SCF and SCF combined, or adriamycin (Figure 4).

**Figure 3:** **Effect of Adriamycin/Anti-SCF on Bcl-2 Expression in MCF-7/AdrRes Cells**. Cell lysates were used to determine the expression of Bcl-2 using ELISA after treatment with the drug adriamycin (D) + SCF, D + anti-SCF, D + SCF + anti-SCF and Drug alone. For each individual experiment data are represented as the mean ± SE of duplicate determinations of 1.25 × 10^4^ cells. ANOVA showed a significant* difference (p < 0.05) between treatments (D) ± SCF and D ± anti-SCF, D ± SCF ± anti-SCF and Drug alone.

**Figure 4:** **Effect of Adriamycin/Anti-SCF on Bcl-2 Expression in MCF-7 Cells**. Cells lysates were used to determine the expression of Bcl-2 using ELISA after treatment with the drug adriamycin (D) + SCF, D + anti-SCF, D + SCF + anti-SCF and Drug alone. For each individual experiment data are represented as the mean ± SE of duplicate determinations of 1.25 × 10^4^ cells. ANOVA showed no significant difference (p > 0.05) between treatments (D) ± SCF, D ± anti-SCF, D ± SCF ± anti-SCF and Drug alone.

### Effect of adriamycin/anti-SCF on annexin V expression in MCF-7/AdrRes and MCF-7 cells

To determine the therapeutic effects of adriamycin, anti-SCF and SCF on annexin V expression, MCF-7 and MCF-7/AdrRes cells were also treated simultaneously for 48 hrs before being examined by ELISA. The expression of annexin V was decreased in MCF-7/AdrRes cells after treatment with adriamycin and SCF, but significantly increased after treatment with adriamycin and anti-SCF (p < 0.042), adriamycin and both SCF and anti-SCF combined and adriamycin alone (Figure 5). There was also a decrease in annexin V expression in MCF-7 cells after treatment with adriamycin and SCF, with a significant increase observed after treatment with adriamycin and anti-SCF (p < 0.001), adriamycin and both anti-SCF and SCF combined and adriamycin alone (Figure 6).

**Figure 5:** **Effect of Adriamycin/Anti-SCF on Annexin V Expression in MCF7/AdrRes Cells**. Cells were used to determine the expression of annexin V using ELISA after treatment with the drug adriamycin (D) + SCF, D + anti-SCF, D + SCF + anti-SCF and Drug alone. For each individual experiment data are represented as the mean ± SE of duplicate determinations of 1.25 × 10^4^ cells. ANOVA showed a significant* difference (p < 0.05) between treatments D ± anti-SCF, D ± SCF ± antiSCF, Drug alone and (D) ± SCF.

**Figure 6:** **Effect of Adriamycin/Anti-SCF on Annexin V Expression in MCF-7 Cells**. Cells were used to determine the expression of annexin V using ELISA after treatment with the drug adriamycin (D) + SCF, D + anti-SCF, D + SCF + anti-SCF and Drug alone. For each individual experiment data are represented as the mean ± SE of duplicate determinations of 1.25 × 10^4^ cells. ANOVA showed a significant* difference (p > 0.05) between treatments D ± anti-SCF, D ± SCF ± antiSCF and Drug alone and (D) ± SCF.

## Discussion

Neoadjuvant chemotherapy is used as a multimodality treatment for breast cancer patients with large and locally advanced disease. One important component of the drug combinations used are anthracyclines (adriamycin), which are given in association with other chemotherapeutic agents such as Taxanes [13]. However, this treatment is compromised by the presence of multidrug resistance (MDR) resulting in treatment failure and subsequent increased morbidity and mortality. Several covariate mechanisms are responsible for multi-drug resistance in breast cancer cells including increased drug efflux (P-glycoprotein-P-gp), CSCs (CD24), drug detoxification (glutathione S-transferase) deregulated apoptosis (Bcl-2 overexpression) and overexpression of cytokines (SCF^)^[8]. The anti-apoptotic expression of Bcl-2 is well documented and its affects on tumourigenic activity [14]. CD24 is a phenotypic surface marker for granulocytes, Bcl’s and CSCs, which are implicated in resistance to both chemotherapy and radiotherapy. Subsequently, some of these progenitor cells differentiate into new mature tumour cells with a chemoresistant phenotype [15]. CSCs were originally described in haematologic malignancies, but this emerging concept is now also applied to solid tumours.

Consequently, there is an increasing need to develop assays which determine the pharmacodynamic effects of both existing and new cancer therapeutics [10]. Annexin V, is a 35 kilodalton (kDa) calcium-dependent protein which binds with high affinity (K = 10-9 M) to phosphatidylserine (PS) residues that are displayed on the outer surface of apoptotic cells [16]. This is not only an alternative non-invasive technique in order to quantify apoptosis and determine pharmacodynamic endpoints after treatment with anti-cancer therapies, but may also be of potential benefit when developing new molecular therapies.

The administration of high-dose chemotherapy facilitated by autologous progenitor cell support such as SCF, the haematopoietic growth factor, is being more frequently applied to the treatment of cancer [17]. In patients with breast and ovarian cancer, lymphoma and multiple myeloma and in conjunction with G-CSF (Granulocyte Colony Stimulating Factor) SCF is used in clinical practice to mobilise CD34+ cells into peripheral blood [18]. In the past SCF expression has been demonstrated in malignant melanomas, pancreatic cancer, glioma cells, gastrointestinal stromal tumours (GIST) and colon cancer [19-23]. Therefore, in preventing chemotherapy induced haematological depression in cancer patients the clinical relevance of SCF and other growth factors or cytokines which may possibly influence tumour proliferation and survival at the level of cancer stem cells, opens questions. Another major concern about this treatment is that SCF may induce protection against chemotherapy in tumour cells that also express the SCF receptor (c-Kit), which has been observed in both haematological and solid cancers. It has been suggested that the maintenance and normal growth of mammary epithelial tissue is influenced by the ckit/SCF pathway with their progressive loss occuring adjacent to malignant transformation [24]. However, one alternative suggestion is that SCF modulates tumour growth and angiogenesis via the involvement of mast cells [25]. Consequently, further examination of the effects of SCF on breast cancer growth and progression is required. Additionally, the activity of anti-SCF may have a multiple role in antagonising the negative growth of breast cancer cells by affecting those pathways involved in CSC and Bcl-2 mediated chemoresistance.

The difference in CD24 expression in MCF-7/AdrRes and MCF-7 cells was demonstrated in this study, and also the ability of anti-SCF to enhance the effects of adriamycin chemotherapy. To the best of our knowledge it is the only study to analyse the synergistic effects of adriamycin and anti-SCF in MCF-7/AdrRes and MCF-7 cells, and their combined effects on Bcl-2-related resistance and annexin V-related cytotoxicity.

Initially, the IC50 minimal dose concentrations obtained from in vitro cytotoxicity assays showed a 1.52 × 10^2^ fold higher resistance to adriamycin in MCF-7/AdrRes cells, compared with MCF-7/WT cells (88.2 μM and 0.579 μM), respectively. In MCF-7/AdrRes cells there was a significant increase in the positivity of CD24 expression compared with a markedly low level in MCF-7 cells. Recently, there have been high levels of CD24 observed in mouse xenografts derived from both CD44+/CD24-/low and CD44+/CD24hi breast cancer cells suggesting important role for CD24 in tumour growth, whilst CD44+/CD24-/low breast cancer cells were not associated with increased tumourigenicity [26]. Further to this, ovarian tumour specimens of a patient showed a sub-population enriched for ovarian CSCs defined by CD24 phenotype. It was observed that the CD24+ sub-population remained quiescent and more chemoresistant compared with the CD24-/low fraction as well as having stem cell-like characteristics such as specific capacity for self-renewal and differentiation. Additionally, CD24 + cells were able to form tumour xenografts in nude mice, whereas equal numbers of CD24- cells did not [27]. Finally, CD24+ cells had lower E-cadherin mRNA levels in comparison to CD24- cells, whilst the mRNA levels of certain stemness genes (Nestin, β-catenin, Bmi-I, Oct4, Oct3/4, Notch1 and Notch4) were more highly expressed.

Interestingly, both adriamycin and SCF combined significantly increased Bcl-2 expression in MCF-7/AdrRes cells, however in MCF-7/WT cells there was no effect. In addition to its cell cycle inhibitory function which markedly increases the cell cycle withdrawal into the G0 quiescent phase Bcl-2 also has the ability to enhance cell survival [28]. This also protects cells from the effects of chemotherapy with increased expression of CD24 being a further contributory factor, modulating not only Bcl-2 expression, but also the presence of CSC populations. The decrease in Bcl-2 expression observed after treatment with both adriamycin and anti-SCF has reduced Bcl-2 related resistance. Subsequently, there were higher annexin V levels observed in MCF-7/AdrRes (and MCF-7/WT cells) after treatment with adriamycin and anti-SCF indicating increased apoptosis, but these were decreased after treatment with adriamycin and SCF. This result differs with our previous study in MCF-7/paclitaxel resistant cells (unpublished data, Jelly et al., 2008). The mechanistic action of each drug combined with anti-SCF may subsequently not only affect Bcl-2 expression, but also the pathways involved in apoptosis leading to annexin V expression, therefore explaining these differences.

Other studies have also reported that Bcl-2 may have distinct biological properties depending on the anticancer agent used when affecting antineoplastic sensitivity [29]. The major advantage of using anti-SCF is that it specifically inhibits SCF and not other key cytokines unlike other generic tyrosine kinase inhibitors such as imatinib, which block several cytokine receptors including c-Kit [30]. In addition there is also the potential when administering this as a combined therapy with adriamycin, to slow the proliferation of normal CD34+ bone marrow cells protecting them from chemotherapy-induced myelosuppression. Also, it may be possible to shorten post-chemotherapy neutropenia. However, normal CD34+ bone marrow cells may become susceptible to cytotoxicity when treating with chemotherapy if anti-SCF reduces Bcl-2 expression [11]. If this combined therapy increases apoptosis in these normal cells of the bone marrow then any therapeutic advantage gained may be lost and therefore further evaluative studies are warranted. In this study it has been demonstrated that Bcl-2 expression is reduced in MCF-7/AdrRes cells after treatment with adriamycin and anti-SCF with annexin V being increased in both MCF-7/AdrRes and MCF-7/WT cells. This possible advantage as well as their cytotoxic effects on normal CD34 + bone marrow cells requires further investigative study. Both adriamycin and anti-SCF combined may potentially improve response to treatment in chemoresistant breast cancer and also improve long term clinical outcome.

## Competing interests

There are no competing interests financial or non-financial (political, personal, religious, ideological, academic, intellectual, commercial or any other) to declare in relation to this manuscript.

## Authors’ contribution

NJ was jointly responsible for the concept, design and completion of all laboratory studies, IH assisted in the laboratory studies. JE and OE participated in the coordination of the study and helped to draft its manuscript. MES was jointly responsible for the concept, design, coordination of the study and also helped to draft its manuscript. All authors read and approved the final manuscript.

## Authors’ information

I. Mr Neil Jelly (NJ) is a PhD student and Lecturer at University of Lincoln.

II. Dr Issam Hussain (IH) is a Lecturer at University of Lincoln

III. Dr Jennifer Eremin (JE) is a Senior Consultant in Medical Oncology

IV. Professor Oleg Eremin (OE) is a Special Professor at the Department of Surgery at Queens Medical Centre, University of Nottingham and Director of Research & Development, Lincoln Hospital

V. Director of the study. Mr. Mohamed El-Sheemy (MES) is a Senior Lecturer at the University of Lincoln & Breast Surgeon at Lincoln Hospital. Director of Clinical Research Laboratory at United Lincolnshire Hospitals NHS Trust

## Funding

Grant from the collaborative Joint Research Fund between University of Lincoln and United Lincolnshire Hospitals NHS Trust.
